RETRACTED

# Sports Enterprise Marketing and Financial Risk Management Based on Decision Tree and Data Mining

**DOI:** 10.1155/2021/7632110

**Published:** 2021-10-15

**Authors:** Yan Zhao

**Affiliations:** School of Philosophy and Public Management, Henan University, Zhengzhou 475001, China

## Abstract

With the development of modern economy, traditional sports industry enterprises have also been further developed in the financial business. How to ensure information security and financial risk management is the problem faced by sports companies. Risk assessment is the use of mathematical models to calculate the risk factors established in the previous step to predict possible risks. In response to the above problems, we developed a sports enterprise marketing and financial risk management model based on decision trees and data mining. First, we have established a relevant evaluation index system and data samples through in-depth understanding of the actual marketing and financial problems of sports companies. Second, we use the decision tree algorithm to mine and explore related data samples and conduct risk assessment through related indicators. By using the model to calculate the probability of occurrence of the risk, analyze the degree of damage. Finally, the algorithm of this paper is analyzed and discussed through simulation experiments.

## 1. Introduction

The development of the financial industry should meet the needs of the real economy. The rise of financial services in the industrial chain of enterprise group finance companies is precisely to ensure that the financial industry serves the real economy [1, 2]. As an internal member of the group, the enterprise group finance company has an incomparable advantage over traditional financial institutions in the development of industrial chain financial services [3]. However, financial business has certain risks. The concept of financial risk management was put forward by Professor Solomon Schobert in the United States in the early twentieth century. Risk management refers to the understanding of event development and the environment, personnel, policies, regulations, and so on [4, 5]. First, we know that risks are everywhere and that risks cannot be eliminated. The purpose of management is to identify potential risk factors and prevent them in the right way [6].

The development of science and technology has promoted the modernization of sports. Advances in technology and engineering have led to an increase in sports achievements. Internet-based games, blogs, and online sports clubs have changed the way sports are observed and applied [7, 8]. Improvements in equipment and tools have spawned new sports such as mountaineering, rock climbing, bungee paragliding, and scuba diving. The innovation of extreme sports has also promoted the development of sports tourism.

RETRACTED

A distinctive feature of entrepreneurs is that they focus on risk management. The rise of financial services in the industrial chain of sports enterprise groups and financial companies is to ensure that the financial industry serves the real economy. There are certain risks in financial business [9]. Risk management refers to the understanding of event development and the environment, personnel, policies, and regulations. The purpose of risk management is to identify potential risk factors and prevent them in the right way. Risk management usually adopts a combination of qualitative and quantitative methods to ensure the safety and normal development of activities and ensure that their economic benefits are not lost [10–12]. Through planned organization, implementation, coordination, and control, sports activities can be carried out in a planned, accurate, orderly, and safe operation. At present, in the literature research on supply chain risk identification, it is found that qualitative research is the main and quantitative research is less [13]. Agrawal and Rautaray [14] described sports risk management as the task of anticipating and regulating threats that have extremely adverse effects on the organization or its capital. It also includes the investigation of organizational processes and the decision-making process to take appropriate action. According to Vesper [15], risk management tasks mean the analysis of financial conditions and the initial perceptions developed from efforts to control productivity and business losses. The development of financial business provides services for the development of the real economy. Risk management usually uses a combination of qualitative and quantitative methods to ensure the safety and normal development of activities and ensure that their economic benefits are not lost [16]. Through planned organization and implementation, coordination and control, and so on, let it proceed in accordance with the preplanned, accurate, orderly, and safe operation. At present, in the literature research on supply chain risk identification, it is found that qualitative research is the main one and quantitative research is less. Tang et al. [16] classified supply chain risks according to the source of the risk and whether the risk is within a controllable range. In the process of supply chain risk identification, Rao further subdivided supply chain risks into external macroenvironmental risks, industry systemic risks, corporate internal risks, and corporate operating risks [17].

RETRACTED

First of all, we know that risks are everywhere, and risks cannot be eliminated. The purpose of management is to identify potential risk factors and prevent them in the right way. Risk assessment is to use mathematical models to calculate the risk factors established in the previous step to predict possible risks. In response to the above problems, we developed a sports enterprise marketing and financial risk management model based on decision trees and data mining. Through in-depth understanding of the actual marketing and financial issues of sports companies, we have established a relevant evaluation index system and data samples. We use decision tree algorithms to mine and explore relevant data samples and conduct risk assessment through relevant indicators. By using the model to calculate the probability of the occurrence of risks and analyze the degree of damage. Finally, the algorithm of this paper is analyzed and discussed through simulation experiments.

## 2. Related Work

### 2.1. Financial Risks

The industrial chain financial services of enterprise group financial companies are playing an increasingly important role in the entire financial service system. However, the time for financial companies of enterprise groups to provide industry chain financial services is relatively short, and there are still many problems in market management, information management, and risk management [18, 19]. A schematic diagram of the financial risk concept of sports companies is shown in Figure 1.

As an emerging financial service, industrial chain financial services have only appeared in China for a short time. Financial company practitioners may be unfamiliar with the business. In the face of unfamiliar businesses, operators often make operational errors after completing a certain number of operators. Circumstances and operational errors caused operational risks [20]. Risk assessment is the use of mathematical models to calculate the risk factors established in the previous step to predict possible risks. By using the model to calculate the probability of risk occurrence, and then analyze the degree of damage. In addition to operating on unfamiliar businesses, irregularities that are prone to occur in the loan approval process will also bring corresponding operational risks [21, 22]. Finance companies that want to develop industry chain finance must first establish an information system. By using the model to calculate the probability of occurrence of the risk, analyze the degree of damage.

### 2.2. Decision Tree

The main methods of data mining include classification, valuation, prediction, association rules, and clustering. Among them, classification, valuation, and prediction belong to guided data mining. These methods can build a model that can describe specific attributes through data. Association rules and cluster analysis are unguided data mining [23, 24]. The schematic diagram of the model structure of the decision tree algorithm is shown in Figure 2.

RETRACTED

This type of method uses all attributes to find a certain relationship. Different data mining methods have their own data mining algorithms, such as decision tree algorithms in classification, regression analysis in prediction, and *K*-means clustering in clustering. Decision tree is one of the well-known machine learning techniques [25, 26]. The purpose of management is to identify potential risk factors and prevent them in the right way. Risk assessment is the use of mathematical models to calculate the risk factors established in the previous step to predict possible risks.

## 3. Sports Enterprise Marketing and Financial Risk Management

The C4.5 and CART algorithms are improvements to the ID3 algorithm. The ID3 algorithm is based on the information gain as the best feature division rule, and the feature with the largest information gain is selected each time during division [26, 27]. The training sample is a key factor that determines the establishment of the decision tree. When there are too few training samples or data problems, the generated decision tree may have abnormal phenomena. This situation will cause the decision tree to be inaccurate and may make the decision tree very complicated [28, 29].

In the multi-index evaluation model, the weight of each index can be distributed in multiple ways. But these methods are roughly divided into two categories. However, these methods are roughly divided into two categories. One is the subjective method, which is an evaluation based on expert experience, including the comparison matrix method and another type of the allocation method is the objective weighting method, which is determined based on the comprehensive evaluation index system, including the direct value method [30, 31]. After the actual creation of the IBM SPSS modeler software and the comparison of the accuracy of the relevant models and the rationality of the partitioning nodes, the most optimized CHAID model is finally selected.

(1) $$\begin{array}{c} \text{CI}=\frac{\lambda_{\max}-n}{n-1}. \end{array}$$

According to research, not all complex and huge decision trees get more accurate rule sets. Therefore, it is necessary to simplify the complex decision tree [32]. The process is called pruning.

(2) $$\begin{array}{c} \text{CR}=\frac{\text{CI}}{\text{RI}}<0.10,\\ M_{i}=\prod_{j=1}^{n}a_{ij},\;i=1,2,\ldots ,n. \end{array}$$

C4.5 is an improvement to the ID3 algorithm, which combines the characteristics of information gain rules and information. This method first finds the attributes with higher information gain rate than the average level from the candidate partition attributes and selects the attribute with the highest gain rate from them. The method used in this article is principal component analysis. The characteristic of this method is to assign weights according to the structural characteristics of the data. The weight of each indicator can fully reflect the contribution of this indicator to the research problem. Therefore, this article uses this method to construct a regional financial risk index.

(3) $$\begin{array}{c} {\bar{W}}_{i}=\sqrt[{n}]{M_{i}}. \end{array}$$

The information gain rate of the attribute to the sample set *D* can be calculated, where IV (*a*) represents the inherent value of feature a, and the more possible values of feature *a*, the greater the value of IV (*a*).

(4) $$\begin{array}{c} W_{i}=\frac{{\bar{W}}_{i}}{\sum_{j=1}^{n}{\bar{W}}_{j}}. \end{array}$$

Therefore, in the candidate attribute set *A*, the attribute with the largest gain rate after division is selected as the best division attribute.  Figure 3 shows a schematic diagram of corporate risk release disturbance data.


(5) $$\begin{array}{c} \lambda_{\max}=\sum_{i=1}^{n}\frac{{\left(AW\right)}_{i}}{nW_{i}}. \end{array}$$

The constraint condition formula is as follows:

(6) $$\begin{array}{c} \left\{\begin{array}{c} \sum_{i=1}^{l}\left(\alpha_{i}-\alpha_{i}^{*}\right)=0\\ \alpha_{i},\alpha_{i}^{*}\in \left[0,C\right] \end{array}\right). \end{array}$$

However, these methods are roughly divided into two categories. One is the subjective method, which is an evaluation based on expert experience, including the comparison matrix method. According to KKT conditions, there are

(7) $$\begin{array}{c} \alpha_{i}\left[\varepsilon +\xi_{i}-y_{i}+w\cdot \varphi \left(x_{i}\right)+b\right]=0. \end{array}$$

The weight of each indicator can fully reflect the contribution of this indicator to the research problem. Therefore, this article uses this method to construct a regional financial risk index. From the above formula, *b* can be obtained as follows:

(8) $$\begin{array}{c} b=\frac{1}{N_{NSV}}\left\{\sum_{0<\alpha_{i}<C}\left[y_{i}-\sum_{x_{i}\in SV}\left(\alpha_{j}-\alpha_{j}^{*}\right)\varphi \left(x_{j}\right)\cdot \varphi \left(x_{i}\right)-\varepsilon \right]+\sum_{0<\alpha_{i}<C}\left[y_{i}-\sum_{x_{j}\in SV}\left(\alpha_{j}-\alpha_{j}^{*}\right)\varphi \left(x_{j}\right)\varphi \left(x_{i}\right)-\varepsilon \right]\right\}. \end{array}$$

The method used in this article is principal component analysis. The characteristic of this method is to assign weights according to the structural characteristics of the data. The purpose of management is to identify potential risk factors and prevent them in the right way. Risk assessment is the use of mathematical models to calculate the risk factors established in the previous step to predict possible risks. When there are too few training samples or data problems, the generated decision tree may have abnormal phenomena. This situation will cause the decision tree to be inaccurate and may make the decision tree very complicated.

RETRACTED

## 4. Actual Case Analysis of Measurement Enterprise Marketing and Financial Risk Management

### 4.1. Test Environment and Data

In the testing process, we divide the input variables into many levels according to the target variables. Combined with the results of corporate marketing tests and questionnaires, the characteristics of large samples, multiple indicators, continuous variables, and categorical variables coexist. After the actual creation of the IBM SPSS modeler software and the comparison of the accuracy of the relevant models and the rationality of the partitioning nodes, the most optimized CHAID model is finally selected.  Figure 4 shows the comparison result of original data and reconstructed data in a financial platform data set.

During the test, the parameters are to be set as the maximum depth of the tree structure is 5 and the minimum number of influencing factor nodes is 100. The minimum number of child nodes is 50, the minimum change value of the Gini coefficient is 0.0001, and the recognition accuracy rate of the 10-layer cross-validation model is used. However, these methods are roughly divided into two categories. One is the subjective method, which is an evaluation based on expert experience, including the comparison matrix method. In the process of supply chain risk identification, Rao further subdivided supply chain risks into external macroenvironmental risks, industry systemic risks, corporate internal risks, and corporate operating risks.  Figure 5 shows the comparison between the original data and the reconstructed data in the data set of a financial analysis institution.

We build model data flow on the IBM SPSS modeler software platform. Tests show that the model performs well in data reconstruction and imitation and can restore risk data well. After the actual creation of the IBM SPSS modeler software and the comparison of the accuracy of the relevant models and the rationality of the partitioning nodes, the most optimized CHAID model is finally selected. After actual measurement, the data output by the model are accurate and reliable and meet the design requirements.

RETRACTED

### 4.2. Quality Analysis of Financial Risk Data Mining

In order to verify the performance of the proposed decision tree model, the decision tree model was compared with some classic classifiers and existing methods. We list the network detection results of the DT-ANN model and some commonly used classifiers. These classifiers are NB (Naive Bayes), LR (logistic regression), SVM (support vector machine), KNN (K nearest neighbor), random forest, decision tree, and ANN (artificial neural network). In this experiment, for ease of comparison, all classifiers are used to process the two data sets listed.  Figure 6 shows the impact of different categories on financial risk testing in the same environment.

We repeated the experiment ten times, and the performance of each model was the average of ten repeated experiments. Different machine learning algorithms were combined to develop hybrid models. In these hybrid models, NB-SVM (category 1) is built on the combination of Naive Bayes classifier and support vector machine classifier. *K*-medics-PNN (category 2) is based on *K*-medics clustering and probabilistic neural network. The hybrid model (category 3) is built based on multiple machine learning algorithms, such as NB, RF, and SVM.  Figure 6 shows that all three categories produce the lowest risk rates (less than 10%). Among the three categories, category 3 which is the combination of NB, RF, and SVM has achieved the lowest risk rate of less than 2%.  Figure 7 shows the impact of financial risk indicators throughput for all three categories in the financial risk testing. It is observed that the proposed model provides reasonable throughput as compared with the other categories of the classifiers.

The table with the largest amount of data in the database is the task table, and the corresponding time of the table related to this table is up to 2 s. The amount of data accessed by general users is small, and the time can be controlled within 0.8 s. Combined with the results of corporate marketing tests and questionnaires, the characteristics of large samples, multiple indicators, continuous variables, and categorical variables coexist. The amount of data that need to be extracted in the report is large, and there are many types of reports, and the time to access various reports is generally within 3 s. Risk assessment is the use of mathematical models to calculate the risk factors established in the previous step to predict possible risks. By using the model to calculate the probability of risk occurrence, and then analyze the degree of damage. In addition to operating on unfamiliar businesses, irregularities that are prone to occur in the loan approval process will also bring corresponding operational risks.  Figure 8 shows the impact of different categories on financial risk testing in the same environment.

RETRACTED

We also tested the system concurrently; that is, multiple users access the system at the same time to operate, and the operation lasts a long time. The main task is to test the task module. When the number of users is less than 50, the CPU usage rate is less than 40%. We compared multiple methods at the same time, and the comparison result is shown in Figure 8. In this experiment, for ease of comparison, all classifiers are used to process the two data sets listed. With the improvement of economic policies and the gradual maturity of financial business, while society is advancing, new business models will inevitably emerge, and corresponding risks will increase. Risk prevention needs to be done to establish more complete risks. In the process of supply chain risk identification, Rao further subdivided supply chain risks into external macroenvironmental risks, industry systemic risks, corporate internal risks, and corporate operating risks.

## 5. Conclusion

When companies solve their own problems through bankruptcy or mergers and acquisitions, this is also a spontaneous risk elimination process, which can effectively prevent the accumulation of financial risks in the nonfinancial corporate sector. The factors affecting the occurrence of regional financial risks have also become complicated, and these complex factors have increased the possibility of regional financial risks. Therefore, a standardized regional financial risk index evaluation system must be established to measure the regional financial risks faced. First of all, we know that risks are everywhere and that risks cannot be eliminated. In the process of supply chain risk identification, Rao further subdivided supply chain risks into external macroenvironmental risks, industry systemic risks, corporate internal risks, and corporate operating risks. The purpose of management is to identify potential risk factors and prevent them in the right way. Risk assessment is the use of mathematical models to calculate the risk factors established in the previous step to predict possible risks.

In response to the above problems, we developed a sports enterprise marketing and financial risk management model based on decision trees and data mining. We have established a relevant evaluation index system and data samples through in-depth understanding of the actual marketing and financial problems of sports companies. We use decision tree algorithms to mine and explore relevant data samples and conduct risk assessments through relevant indicators. By using the model to calculate the probability of occurrence of the risk, analyze the degree of damage. Finally, the algorithm of this paper is analyzed and discussed through simulation experiments.

RETRACTED

## Figures and Tables

**Figure 1:** Schematic diagram of the financial risk concept of sports companies.

**Figure 2:** Schematic diagram of the model structure of the decision tree algorithm.

**Figure 3:** Schematic diagram of corporate risk release disturbance data.

**Figure 4:** Comparison of original data and reconstructed data in a financial platform data set.

**Figure 5:** Comparison of original data and reconstructed data in a data center of a financial analysis institution.

**Figure 6:** The impact of different categories on financial risk testing in the same environment.

**Figure 7:** The impact of different environments in the same category on financial risk testing.

**Figure 8:** Comparison of financial risk data mining effects of different experimental methods.

## Data Availability

The data used to support the findings of this study are included in the article.
